# Lymphoepithelial-like carcinoma of the parotid gland: a case report and a brief review of the western literature

**DOI:** 10.1186/1746-1596-8-115

**Published:** 2013-07-15

**Authors:** Maria R Ambrosio, Maria G Mastrogiulio, Aurora Barone, Bruno J Rocca, Carmine Gallo, Stefano Lazzi, Lorenzo Leoncini, Cristiana Bellan

**Affiliations:** 1 Department of Medical Biotechnology, Pathological Anatomy Section, University of Siena, via delle Scotte, Siena 6-53100, Italy; 2 Department of Biomedical and Neuromotor Sciences, Section of Anatomic Pathology, “M.Malpighi”, Bellaria Hospital, University of Bologna, Bologna, Italy

## Abstract

**Background:**

Primary lymphoepithelial-like carcinoma of the parotid gland is a rare tumour with an increased incidence among Eskimos and Orientals. In these populations, it is usually associated with Epstein-Barr virus. In Western countries, salivary gland lymphoepithelial-like carcinomas are uncommon and only 14 cases have been described so far; among these, only five cases showed Epstein-Barr virus positivity.

**Case report:**

A 45-year-old woman was admitted to Siena Hospital for evaluation of a pre-existent (2 years) painless and tender submandibular mass, rapidly enlarging since two months. On physical examination, a 2.5-cm mass was found in the right parotid. It was firm, mobile and non-tender. Laboratory data were within reference range. Nuclear magnetic resonance detected a 2,5×1,5×1-cm well-circumscribed mass in the deep lobe of the right parotid. A total right paroditectomy with dissection of a satellite lymph node was performed. On the basis of morphological, immunohistochemical and molecular biology findings, a diagnosis of stage II (according to TNM7) Epstein Barr-virus positive, undifferentiated lymphoepithelial-like carcinoma of the parotid gland was made. Twenty months after surgery the patient was free of disease.

**Conclusions:**

Further studies seem to be necessary to completely elucidate the oncogenic role of Epstein Barr-virus in these tumors, which have identical morphology but different prognosis and variable presence of the virus.

**Virtual Slides:**

The virtual slide(s) for this article can be found here: http://www.diagnosticpathology.diagnomx.eu/vs/1260381551000616

## Background

Salivary gland neoplasms comprise less than 3% of all neoplasms in the head and neck region [1]. Eighty percent occur in the parotid gland, of which approximately 80% are benign and 20% are malignant [2]. An exception is represented by the Eskimo population, in which 60% of the parotid gland tumors are malignant, the majority being lymphoepithelial-like carcinoma (LELC) [3]. LELC is analogous to lymphoepithelial carcinoma (LE) of the nasopharynx which is very common among Southern China inhabitants [1]. LE is a poorly differentiated carcinoma composed of sheets of large atypical epithelial cells intermingled with a benign inflammatory infiltrate that is rich in lymphocytes and plasma cells. It is equivalent to type 3 nasopharyngeal carcinoma according to the World Health Organization (WHO) classification [4]. A consistent feature is the association of this type of carcinoma with Epstein-Barr virus (EBV), which is detectable in all tumour cells [5]. LELC has the same histological patterns as undifferentiated LE and is associated with a variable amount of lymphoid infiltrate in the stroma. However, LELC arises in organs other than nasopharynx, including larynx [6], tonsils [7], salivary glands [8], lung [9], thymus [10], stomach and duodenum [11], breast [12], renal pelvis and urinary bladder [13], uterine cervix [14], endometrium [15-17] ovary [18,19], vulva and vagina [20-22]. EBV is detected in LELCs arising in organs of foregut derivation and in Asian women but rarely in LELCs of other sites or in non-Asian patients [6-22]. When the tumors occur in the salivary glands, the parotid gland is more often involved [23]. Women are affected more than men with an average age of 40 years (range: 20–60 years) [24]. Two thirds of LELC arise *de novo*, whereas the remaining develop in the setting of a preceding or concurrent benign lymphoepithelial lesion [25]. To the best of our knowledge, 14 cases [1,4,25-32] of this unusual cancer occurring in the salivary glands have been described in Western population and only in five cases EBV encoded RNAs (EBER) was positive [26-28]. Herein, we present the sixth case associated with EBV infection and the first one showing LMP-1 positivity.

## Case presentation

### Ethics Statement

Ethics approval for this study was obtained from the Institutional Review Board at the University of Siena (Italy).

### Clinical summary

A 45-year-old woman was admitted to Siena University Hospital for evaluation of a pre-existent (2 years) painless and tender submandibular mass, rapidly enlarging since two months. She denied any history of facial weakness, cervical lymphadenopathy, or recent fever, tooth extraction or trauma. Her medical and family history was unremarkable. On physical examination, a 2.5-cm mass was found in the right parotid. It was firm, mobile and non-tender. Facial nerve function was intact and no enlarged cervical lymph node or other masses were palpated. Examination of the nasopharynx and Waldeyer’s ring by nasopharingoscopy found no lesions. Laboratory data were within reference range. Nuclear magnetic resonance (NMR) detected a 2,5×1,5×1-cm well-circumscribed mass in the deep lobe of the right parotid. A total right paroditectomy with dissection of a satellite lymph node was performed.

### Pathologic findings

At gross examination, the parotid gland appeared almost entirely substituted by a yellowish white, firm and multinodular lesion measuring 2.5×1.6×1.2 cm. Macroscopically, the tumor did not involve surgical margins. Representative sections of the surgical specimen were performed, routinely processed, stained with haematoxylin and eosin and examined by light microscopy. Microscopically, solid carcinomatous sheets, trabeculae and isolated small groups of neoplastic epithelial cells intermingled with lymphoid tissue and surrounded by fibrous tissue were observed [Figure 1A]. The carcinomatous areas were sometimes characterized by crowded and overlapping syncitial-appearing large tumor cells with scant amphophilic cytoplasm and vesicular haphazardly arranged nuclei [Figure 1B]. Nuclei had diameters up to 8 times the diameter of lymphocyte nuclei and sharply demarcated nuclear rims, finely speckled chromatin and prominent, usually single, eosinophilic nucleoli. There were nuclear atypia and numerous mitotic figures [Figure 1C]. Minute areas of coagulative necrosis were present. The lymphoid infiltrate was composed mainly of small lymphocytes and, in some areas, formed follicular structures with germinal centers. The density of lymphoid tissue varied from areas with a few lymphocytes and plasma cells in between carcinomatous islands or accompanying carcinomatous trabeculae to areas where abundant lymphoid cells broke the tumor islands into small groups of cells. The surrounding parotid tissue contained foci of chronic sialoadenitis and scattered benign lymphoepithelial lesion. The satellite lymph node showed no infiltration by the tumor.

**Figure 1:** **Histopathological characteristics of the LELC of the parotid gland.** (**A**) Isolated small groups of carcinomatous cells (arrows) are immersed in an abundant lymphoid tissue. (**B**) The neoplastic sheets are composed of syncytial-like cells. (**C**) Nuclear atypia and numerous mitotic figure are observed. [**A-C** Haematoxylin-Eosin (H&E). A, Original Magnification (O.M.): 5x; B, O.M.: 10x; C, O.M.: 20x].

Immunohistochemistry analysis showed that the carcinomatous cells were decorated by cytokeratin 7, LMP-1 and Fascin [Figure 2A-C] as well as by vimentin, whereas they were negative for cytokeratin 20 and lymphoid markers. The proliferation index (Mib-1) was about 80%. The lymphoid tissue contained a mixture of T cells (CD3 positive) (Figure 3A) and B cells (CD20 positive) (Figure 3B) and follicles with CD10-positive germinal centers. Numerous CD30 positive blasts were present. EBER-positive signals were observed in both the carcinomatous and lymphoid cells (Figure 3C).

**Figure 2:** **Immunohistochemichal analysis of the carcinomatous component of the lesion.** Carcinomatous sheets showed positivity to (**A**) CK20, (**B**) LMP-1 and (**C**) fascin. (**A**, O.M.: 10x; **B** and **C**, O.M.: 40x).

**Figure 3:** **Immunohistochemichal analysis of the lymphoid component of the lesion.** Lymphoid cells were (**A**) CD3 positive and (**B**) CD20 positive. (**C**) EBER positive signals were observed in both carcinomatous and lymphoid areas (A and C, O.M.: 20x; B, O.M.: 10x).

On the basis of morphological, immunohistochemical and molecular biology findings, a diagnosis of stage II (according to TNM7) EBV-positive, undifferentiated LELC of the parotid gland was made. Twenty months after surgery the patient is free of disease, as confirmed by NMR.

## Discussion

The term *lymphoepithelioma* was introduced in 1921 to refer to an undifferentiated carcinoma of the nasopharynx with a dense lymphocytic component [33]. It is characterized by nests of undifferentiated epithelial cells infiltrated by a prominent benign reactive lymphocytic infiltrate. Epstein-Barr virus is frequently present in the malignant epithelial cells of this carcinoma [17]. Such association was first reported by Harold Zur Hausen in 1970 [19]. LELC is a subtype of poorly differentiated squamous cell carcinoma, identical to the LE described in the nasopharynx but originating in other anatomic sites. Most of the reported cases of primary LELC of the salivary gland occurred in Asians and Eskimos whereas they are uncommon in Americans and Europeans [26]. To the best of our knowledge, 14 cases have been previously described in western people [1,4,25-32]. All lesions affected parotid gland. The median age of the patients was 54,6 years (range: 32–74), with a female predominance (78.5%). Six patients (43%) showed lymph node metastasis (not all data available). Only two patient (14%) received radiation therapy alone, the others being treated by total parotidectomy with or without postoperative radiation therapy. All the patients were alive at the last follow-up (not all data available). *In situ* hybridization for EBV was positive only in 5 patients (36%, not all data available). Clinico-pathological and therapy data of all these 14 cases are listed in Table 1.

**Table 1:** Clinicopathological features of patients with LELC of the parotid gland described in the Western literature

**Author**	**Sex**	**Age**	**Treatment**	**Clinical outcome**	**EBER**	**Other data**
Ferlito A, 1977 [30]	F	36	SP	At the last follow-up, no signs of relapse	n.a.	Cervical lymph node metastasis
Ferlito A, 1977 [30]	F	55	SP	At the last follow-up, no signs of relapse	n.a.	n.a.
Ferlito A, 1977 [30]	F	32	RP	At the last follow-up, no signs of relapse	n.a.	n.a.
Kott ET, 1984 [31]	M	51	RT	At 11-year follow-up, no signs of relapse	n.a.	Cervical lymph node metastasis
Kott ET, 1984 [31]	F	42	SP + RT	At 12-month follow-up, no signs of relapse	n.a.	n.a.
Kountakis Se,1995 [1]	F	68	SP + RT	At 24-month follow-up, no signs of relapse	negative	Metastasis to intraparotid lymph node
Kountakis Se, 1995 [1]	F	57	RP + RT	At 24-month follow-up, no signs of relapse	negative	Lymph node metastasis
Kotsianti A, 1996 [32]	M	64	SP	At the last follow-up, no signs of relapse	positive	Regional lymph node metastasis
Squillaci S, 2000 [27]	F	45	SP + RT	At 15-month follow-up, no signs of relapse	positive	n.a.
Wu DL, 2001 [26]	F	54	RP + RT	At 24-month follow-up, no signs of relapse	positive	n.a.
Squillaci S, 2002 [4]	F	72	SP + RT	At 36-month follow-up, no signs of relapse	positive	Periparotid lymph node metastasis
Bialas M, 2002 [28]	F	74	RT	n.a.	positive	n.a.
Ayache S, 2004 [25]	M	47	RP + RT	At 7-month follow-up, no signs of relapse	negative	Neural metastasis
Manganaris A, 2007 [29]	F	67	SP + RT	At 12-month follow-up, no signs of relapse	n.a.	n.a.

*RP* radical parotidectomy, *SP* superficial parotidectomy, *RT* radiotherapy, *n.a.* not available.

The origin and pathogenesis of LELC is still unknown [1]. It is thought to arise in either of two settings: malignant transformation of a myoepithelial island or malignant transformation of glandular and ductal inclusions in intraparotid lymph node. The association with EBV has suggested a possible role for the virus in the etiology but the relationship is controversial, considering that some LELC at specific anatomical sites have never been proven to be associated with EBV [17]. There is no satisfactory explanation for EBV being commonly present in certain anatomic sites, but not in others. In the past, it was believed that only foregut-derived organs (salivary gland, stomach, thymus, and lung) were susceptible to EBV-associated carcinogenesis, perhaps because these organs are in close proximity to sites of natural viral replication [19]. The portal of entry of the virus is thought to be the oropharyngeal mucosa, which also serves as the site of production of the virus, which is periodically shed in saliva [27]. The infection of lymphocytes permits systemic dissemination, and following primary infection, EBV lies latent in a few lymphocytes for the duration of life. The establishment of a persistent infection protects the virus against the immune response. Thus, EBV can immortalize human keratinocytes promoting neoplastic transformation. The oncogenic role of EBV is elicited by its products. Among these, LMP-1 has a driving role. Expression of LMP-1 prevents apoptosis, induces abnormal cell proliferation, deregulates epithelial growths and inhibits differentiation, with the epithelial cells showing the features of transformed cells [34]. However, the expression of this protein was observed only in few EBV-linked salivary LELC from Asian patients and our case is the first one in which LMP-1 positivity was detected in a Western patient. These findings may suggest that different strains of EBV could be involved in the pathogenesis of salivary LELC in different geographic areas. These strands may express LMP-1 with different genetic sequence and thus different immunohistochemical positivity [35]. A recent study has reported the immunoreactivity of LELC neoplastic cells for fascin as in our case [4]. Fascin is a 55 Kda globular protein that is expressed in almost all cellular types. It acts organizing actin-based structures (i.e. filopodia, microspikes and lamellipodial ribs), and cytoplasmic microfilament bundles [36,37]. In addition fascin packs F-actin into parallel bundles. The association of fascin with F-actin is strongly regulated by the extracellular matrix (ECM) environment of cells and is required for cell migration [38,39]. It is possible that latent EBV infection of epithelial salivary gland cells can upregulate transcriptional activity of the fascin-1 gene with increased synthesis of the protein in cytoplasm. This phenomenon could play an important role in the progression to an invasive phenotype of transformed cells, with the loss of cell to cell adhesion and loss of junctional communications. Furthermore, fascin-positive stromal dentritic cells might be modified by functional changes via the EBV induced release of soluble CD83 with inhibition of stimulation of T-cell proliferation [39]. However, the absence of EBV genome in most LELC cases [19] implies that EBV is not a necessary factor in the aetiology or pathogenesis of LELC, and that genetic, environmental or geographic factors may be involved [17].

Differential diagnosis of LELC include squamous and mucoepidermoid carcinoma with abundant lymphocytic infiltration, poorly differentiated large cell carcinoma of salivary origin, and nasopharyngeal carcinoma with parotid extension. The first three entities are easily distinguished from LELC by histology. Otherwise, nasopharyngeal carcinoma can be difficult to differentiated and requires a complete clinical, radiological, morphological and immunohistochemical evaluation [27].

## Conclusion

We presented a case of EBV-positive LELC of the parotid gland with a brief review of the literature. On the basis of our findings, further studies seem to be necessary to completely elucidate the oncogenic role of EBV in these tumors, which have identical morphology of nasopharyngeal LE but different prognosis and variable presence of the virus. When stratified according to stage, LELC has a more favorable outcome. This is probably due to the presence of prominent lymphoid tissue, which may represent a host response against the tumour, and to its biological characteristics, including responsiveness to radiotherapy. Biologic significance of EBV in LELC is unclear as well as its prognostic importance because of relatively small numbers of cases and short follow-up [17].

As previous studies demonstrated that fascin is a downstream mediator of LELC carcinogenesis, it may represent a molecular target for therapeutic intervention [4]. An analysis of additional cases with long-term follow-up as well as systematic evaluation of fascin expression would be necessary to shed new light on the pathogenesis of this rare and challenging tumour.

### Consent

Written informed consent was obtained from the patient for publication of this Case Report and any all accompanying images. A copy of the written consent is available for review by the Editor-in-Chief of this journal.

## Abbreviations

LELC: Lymphoepithelial-like carcinoma; LE: Lymphoepithelial carcinoma; EBV: Epstein-Barr virus; NMR: Nuclear magnetic resonance; EBER: Epstein-Barr virus encoded RNA.

## Competing interest

The authors declare that they have no competing interests.

## Authors’ contributions

MRA wrote the paper; MGM and BJR performed analysis of the histological sections; AB carried out the immunoassays; SL made contributions to acquisition of clinical data; CG gave tools; LL contributed his expertise in the field and fruitful discussion; CB coordinated the work and gave final approval of the version to be published. All authors read and approved the final manuscript.

## References

[B1] KountakisSESooHooWMaillardA**Lymphoepithelial carcinoma of the parotid gland**Head and Neck19951744545010.1002/hed.28801705168522448

[B2] SkolnikEMFreidmanMBeckerSTumors of the major salivary glandsLaryngoscope19778784386119413010.1288/00005537-197706000-00001

[B3] NielsenNHMikkelsenFHanseJPIncidence of salivary gland neoplasm in Greenland with special reference to an anaplastic carcinomaActa Pathol Microbiol Scand19788618519310.1111/j.1699-0463.1978.tb02030.x696318

[B4] SqullaciSConstantine SULymphoepithelioma-Like Carcinoma (LELC) of Salivar Gland Associated with Epstein-Barr Virus in a North Italian Woman. Report of a New Case and Review of the LiteratureNew Developments in Epstein-Barr Virus Research2006New York: Nova Science Publishers, Inc233260

[B5] JangSJPaikSSLeeWMLymphoepithelial Carcinoma of the Submandibular GlandJKMS19971225225510.3346/jkms.1997.12.3.252PMC30542929250924

[B6] SoneMNakashimaTNagasakaTLymphoepithelioma-like carcinoma of the larynx associated with an Epstein-Barr viral infectionOtolaryngol Head Neck Surg1998191347967452710.1016/S0194-5998(98)70185-8

[B7] KlijanienkoJMicheauCAzliNUndifferentiated carcinoma of nasopharyngeal type of tonsilOtolaryngol Head Neck Surg1989115731410.1001/archotol.1989.018603000850232541744

[B8] LeungSYChungLPYuenSTLymphoepithelial carcinoma of the salivary gland: in situ detection of Epstein-Barr virusJ Clin Pathol1995481022710.1136/jcp.48.11.10228543624PMC503007

[B9] CastroCYOstrowskiMLBarriosR**Relationship between Epstei-Barr virus and lymphoepithelioma-like carcinoma of the lung**: **a clinicopathologic study of 6 cases and review of the literature**Hum Pathol2001328637210.1053/hupa.2001.2645711521232

[B10] WichMRScheitauerBWWeilandLHPrimary thymic carcinomasAm J Surg Pathol198266133010.1097/00000478-198210000-000036295194

[B11] ShoushaSLuqmaniYAEpstein-Barr virus in gastric carcinoma and adjacent normal gastric and duodenal mucosaJ Clin Pathol19944769569810.1136/jcp.47.8.6957962618PMC502138

[B12] DadmaneshFPeterseJLSapinoALymphoepithelioma-like carcinoma of the breast: lack of evidence of Epstein-Barr virus infectionHistopathology200138546110.1046/j.1365-2559.2001.01055.x11135047

[B13] AminMBRoJYLeeKMLymphoepithelioma-like carcinoma of the urinary bladderAm J Surg Patho1994184667310.1097/00000478-199405000-000058172321

[B14] MillsSEAustinMBRandallMELymphoepithelioma-like carcinoma of the uterine cervix. A distinctive, undifferentiated carcinoma with inflammatory stromaAm J Surg Pathol19859883910.1097/00000478-198512000-000043934992

[B15] VargasMPMerinoMJLymphoepithelioma-like carcinoma: an unusual variant of endometrial cancer: a report of two casesInt J Gynecol Pathol19981727227610.1097/00004347-199807000-000139656125

[B16] RahimiSLenaAVittoriGEndometrial lymphoepithelioma-like carcinoma: absence of Epstein-Barr virus genomesInt J Gynecol Pathol200717532510.1111/j.1525-1438.2007.00793.x17362326

[B17] AmbrosioMRRoccaBJMourmourasVLymphoepithelioma-like carcinoma of the endometriumPathologica2010102576123596758

[B18] LeeSParkSYHongEKLymphoepithelioma-like carcinoma of the ovaryArch Pathol Lab Med2007131171581797949210.5858/2007-131-1715-LCOTOA

[B19] AmbrosioMRRoccaBJOnoratiMLymphoepithelioma- like carcinoma of the ovaryInt Surg Pathol201119514710.1177/106689690935433620444729

[B20] AxelsenSMStampIMLymphoepithelioma-like carcinoma of the vulvar regionHistopathology19952728128310.1111/j.1365-2559.1995.tb00222.x8522294

[B21] BosmullerHHaitchi-PetnehazySGruberCLymphoepithelioma-like carcinoma of the vulva, an underrecognized entity? Case report with a single inguinal micrometastasis detected by sentinel node techniqueDiagn Pathol20116410.1186/1746-1596-6-421219641PMC3023728

[B22] DietlJHomyHPKaiserlingELymphoepithelioma-like carcinoma of the vagina: a case report with special reference to the immunophenotype of the tumor cells ant tumor-infiltrating lymphoreticular cellsInt J Gynecol Pathol199413186910.1097/00004347-199404000-000138005741

[B23] KuoTHsuehCLymphoepithelioma-like salivary gland carcinoma in Taiwan: a clinicopathological study of nine cases demonstrating a strong association with Epstein-Barr virusHistopathology199731758210.1046/j.1365-2559.1997.5830814.x9253628

[B24] MradKBrahimEBDrissMLymphoepithelioma-like carcinoma of the submandibular salivary gland associated with Epstein- Barr virus in a North African womanVirhows Arch200444541942010.1007/s00428-004-1072-715258757

[B25] AyacheSChatelainDPerretCLe carcinoma Lymphoepithelial de la parotide: une tumeur rare chez un patient europeenLaryngol Otol Rhinol2004125423924115712695

[B26] WuDLShemenLBradyTMalignant lymphoepithelial lesion of the parotid gland: a case report and review of the literatureEar Nose Throat J20018011803611816892

[B27] SquillaciSBertalodGVagoLLymphoepithelioma-like carcinoma of the parotid *gland.* Description of a case with detection of EBV by in situ hybridizationPathologica20009218919410902430

[B28] BiałasMSińczakAChoińska-StefańskaAEBV-positive lymphoepithelial carcinoma of salivary gland in a woman of a non-endemic area-a case reportPol J Pathol2002534235812597342

[B29] ManganarisAPatakioutaFXirouPLymphoepithelial carcinoma of the parotid gland: is an association with Epstein-Barr virus possible in non-endemic areas?Int JOral Maxillofac Surg20073655655910.1016/j.ijom.2006.12.01217306504

[B30] FerlitoAFiore DonatiLMalignant lymphoepithelial lesions’ (undifferentiated ductal carcinomas of the parotid gland). Three case reports and review of the literatureJ Laryngol Otol1977911086988310.1017/S0022215100084498336820

[B31] KottEGoepfertHAyalaALymphoepithelial carcinoma (Malignant Lymphoepithelial Lesion) of the Salivary GlandsArc Otolaryngol1984110505310.1001/archotol.1984.008002700540146689908

[B32] KotsiantiACostopolosJMorgelloSUndifferentiated carcinoma of the parotid gland in a white patient: detection of Epstein-Barr virus by in situ hybridizationHum Pathol1996271879010.1016/S0046-8177(96)90144-68543318

[B33] AnagnostopoulosIHummelMEpstein-Barr virus in tumoursHistopathology19962929731510.1111/j.1365-2559.1996.tb01414.x8910038

[B34] LuSYHuangCCHsiungCYPrimary lymphoepithelioma-like carcinoma of minor salivary gland: a case report with immunohistochemical and in situ hybridization studiesHead Neck20062818218610.1002/hed.2031216240326

[B35] JenKYChengJLiJMutational events in *LMP1* gene of Epstein-Barr virus in salivary gland lymphoepithelial carcinomasInt J Cancer200310565466010.1002/ijc.1110012740914

[B36] AdamsJCRoles of fascin in cell adhesion and mobilityCurr Opin Cell Biol20041659059610.1016/j.ceb.2004.07.00915363811

[B37] KureishyNSapountziVPragSFascins, and their roles in cell structure and functionBioessays20022435036110.1002/bies.1007011948621

[B38] AnilkumarNParsonsMMonkRInteraction of fascin and protein Kinase C-alfa: a novel intersection in cell adhesion and motilityEMBO J2003225390540210.1093/emboj/cdg52114532112PMC213775

[B39] KotzorNLechmannMZinserEThe soluble form of CD83 dramatically changes the cytoskeleton of dentritic cellsImmunobiology200420912914010.1016/j.imbio.2004.04.00315481147

